# Fostering Advocacy Behavior of Employees: A Corporate Social Responsibility Perspective From the Hospitality Sector

**DOI:** 10.3389/fpsyg.2022.865021

**Published:** 2022-04-27

**Authors:** Naveed Ahmad, Zia Ullah, Esra AlDhaen, Heesup Han, Antonio Ariza-Montes, Alejandro Vega-Muñoz

**Affiliations:** ^1^Faculty of Management Studies, University of Central Punjab, Lahore, Pakistan; ^2^Faculty of Management, Virtual University of Pakistan, Lahore, Pakistan; ^3^Faculty of Business Administration, Lahore Leads University, Lahore, Pakistan; ^4^Marketing Department, College of Business and Finance, Ahlia University, Manama, Bahrain; ^5^College of Hospitality and Tourism Management, Sejong University, Seoul, South Korea; ^6^Social Matters Research Group, Universidad Loyola Andalucía, Córdoba, Spain; ^7^Public Policy Observatory, Universidad Autónoma de Chile, Santiago, Chile

**Keywords:** corporate social responsibility, advocacy behavior, engagement, hotel sector, sustainability

## Abstract

Considering the stiff competitiveness situation in every sector, promoting the advocacy behavior of employees is of seminal importance for an organization. With this regard, the hospitality sector has no exceptions, however, a review of the prior literature uncovers that most of the prior studies on advocacy behavior were conducted from the standpoint of consumers, and the role of employees’ advocacy behavior, especially in the context of the hospitality sector, remained an understudied area. Research also shows that the corporate social responsibility (CSR) efforts of an organization can significantly influence employees’ behavior but the relationship of CSR to spur employees’ advocacy behavior was not discussed earlier. Against this knowledge gap, the current work aims to investigate the relationship between CSR and employees’ advocacy behavior in the hotel sector of a developing economy with the mediating effect of employees’ engagement. A hypothesized model was developed, which was validated by collecting data from different hotel employees through a self-administered questionnaire. The findings offer different theoretical and practical implications. Theoretically, one important implication was that the CSR perceptions of hotel employees can drive their advocacy behavior. Practically, the study implicates that hotels can improve their reputation significantly by converting their employees into advocates, as the personal information source is preferred over company-generated information sources. Moreover, the CSR commitment of a hotel can lead the employees to a higher level of engagement, which then motivates them to act as advocates.

## Introduction

With the rise of globalization and information technology, the competitive landscape is changing continuously in every sector than ever before. In the current era of stiff competition, contemporary organizations are searching for different ways to survive and outperform their rivals. In this aspect, the behavior of employees in an organization has been reported as a critical enabler for the success of a business (Imamoglu et al., 2019; Clack, 2020). Generally, it is established that professional behavior develops a collaborative work environment, which boosts the business operations, and concurrently leads an organization toward success. Perhaps, this is why employees’ role in the workplace has become a contemporary topic of academic debate (Siyal et al., 2020). Given that the role of employees is seminal for the success of an organization, irrespective of its size and sector, employee advocacy behavior has been receiving mounting importance recently (Men and Yue, 2019; Thelen, 2020). The underlying reason for organizational interest in employee advocacy behavior lies in the fact of high level of trust that individuals confer to personal sources of information rather than relying on the organizational sources of communication like an advertisement and others (Murray, 1991). Buttressing this, a report by The Nielsen Group indicated that 83% of respondents from 60 countries trust the information and recommendations they receive from personal sources (McCaskill, 2015). Moreover, research shows that the interest of organizations to foster employee advocacy has raised significantly during the past years (Terpening et al., 2015). Responding to this, Jason Frank, the CEO of MSL-Group, posited that the employees have been emerging as the ultimate reputation builders for an organization, where an organization sells its experiences instead of product or services, and where the truth is shared by the insiders (the employees; Frank, 2015). In spite of the mounting importance of employee advocacy behavior, research in this area is still limited (Men, 2014). Given that the prior research studies have primarily focused on the advocacy behavior of consumers (Chelminski and Coulter, 2011; Jayasimha and Billore, 2016), there is a need to carry out more research in this area from the perspective of employees. Moreover, what could be the factors that can spur the advocacy behavior of employees is also a less explored terrain.

In this regard, research shows that employees’ corporate social responsibility (CSR) perceptions can be positively linked with their attitudinal and behavioral intentions (Farooq et al., 2014; Mi et al., 2018). For example, it was mentioned in the prior literature that CSR could foster employees’ pro-environmental behavior (Molnár et al., 2021; Yu et al., 2021), innovative behavior (Ahmad et al., 2021), citizenship behavior (Zhao and Zhou, 2021), and job crafting (Hur et al., 2021). Despite these recent contributions, little is known about the relationship between CSR and employees’ advocacy behavior. There have been some recent contributions in this vein (Castro-González et al., 2019; Xie et al., 2019), these researches were conducted from a consumer perspective and neglected employees’ perspective. Therefore, one of the prime objectives of the current work is to investigate the relationship between CSR and employees’ advocacy behavior.

When it comes to employees’ behavior, it was found that organizational and personal factors shape behavior. Where, at the level of organization, CSR can influence the positive psychology of employees, at a personal level, employees engagement is attributed to guiding the behavior of employees in a workplace (Kang and Sung, 2017; Sun and Bunchapattanasakda, 2019). At the same time, different studies also reported that CSR is an enabler of employee engagement (Duthler and Dhanesh, 2018). Specifically, in a plethora of studies, the mediating role of employee engagement, as an outcome of CSR, was reported (Chaudhary and Akhouri, 2018b; Ali et al., 2020). However, such mediating role of employee engagement between CSR and employees’ advocacy behavior was barely explored previously. Therefore, another objective of this analysis is to test the mediating effect of employee engagement between CSR and employees’ advocacy behavior relationship.

The current work tends to fill the following knowledge gaps. First, the current work aims to test the association of CSR and employee advocacy behavior with the mediating role of employees’ engagement in a unified model. Second, the current work attempts to advance the field of organizational management by promoting advocacy behavior among employees as an outcome of CSR. As mentioned earlier in this draft, the topic of advocacy behavior largely remained an area of investigation for consumer behavior research. Third, the current work offers a unique contribution to the literature of hospitality management, especially the hotel sector. Given that this sector has been largely reported for its high employee turnover (Glenn, 2016; Erica, 2019; Amanda, 2020), and stiff rivalry, the current work attempts to help this sector by proposing CSR for a win-win strategy by fostering employees’ engagement and advocacy behavior. Last, the current work aims to advance the literature from a developing economy perspective (Pakistan). In this regard, most CSR and employee management research, especially in the hospitality sector, was carried out in developed countries (Appiah, 2019; Kim et al., 2020). The rest of the current draft is divided into different sections for the convenience of the readers. For instance, the upcoming section deals with theoretical underpinning and related literature to formulate the hypotheses. The next section describes the methodology, where the authors provide the information about population, sample, and the data collection process. The fourth section deals with results and analysis to validate the hypotheses. Lastly, in the discussion section, the authors provide a discussion of their results in relevance to previous studies. Moreover, this section also includes implications, limitations, and conclusions.

## Literature Review

The hypothesized framework of the current analysis is underpinned in the theory of social identity. Originally proposed by Tajfel (1978), this theory has largely been employed in several behavioral studies (Shen et al., 2018; Cruwys et al., 2020). Indeed, the theory of social identity posits that an individual’s behavior (the employees in the current context) is largely influenced by his self-concept about a social group (here, social group means an organization) to which he identifies himself. To elucidate further, based on some social characteristics, which are in congruence with an individual’s personal values, of a social group, the individuals strongly identify with that group. Thus, the process of social identification builds a strong social bond between a social group and its members. Buttressing this to the current context, the CSR philosophy of an organization is perceived by employees as a social benefit for all stakeholders (consumers, employees, community, and even creditors), thus this social character of a socially responsible organization is expected to build a social bond between employees and the organization. Once social bonding is created as an outcome of CSR, each group member is self-motivated to put forth every effort that can benefit the group’s overall performance. Thus, in response to the CSR efforts of an organization, the employees are expected to become the advocates, who then consider the organization as their own organization. All this process improves their engagement with the organization and urges them to make every effort to enhance the organization’s overall performance. Therefore, the authors of the current draft feel this theory provides a logical explanation for the hypothesized framework of the current study.

### Defining Employee Advocacy and Relating It With CSR

Given that the field of employee advocacy is still in its formative stages, there is no available universal definition of this concept. The work of Božac et al. (2017) relates it with the promotion of an organization by the employees. In like vein, Schweitzer and Lyons (2008) define employee advocacy as an act of employees to work as part-time marketers to promote the organization to potential consumers and employees. Another definition of employee advocacy (which is applied here too) was provided by Men (2014) who argued that “it is a behavioral construct that is entirely voluntary in its nature and the employees under this philosophy act not only as of the promoters but also as defenders for their organization, its product and services and its brand to the external community.” When linked to the current work’s context, as employee advocacy behavior is a voluntary commitment of employees with their organization, such volunteer commitment can be well linked with the CSR orientation (a voluntary organizational commitment) of an organization. This viewpoint can be seen in the seminal work of Dewhurst et al. (2009) and Kremer et al. (2019) who documented that CSR perception of employees can be well linked with their extra-role (voluntary) performance rather than to foster their bottom line performance. Moreover, the literature also states that the act of employee advocacy has several similarities with the concept of organizational citizenship behavior (OCB), which is also voluntary and is not assumed to be rewarded by the organization explicitly (Walden and Westerman, 2018). When looked from this perspective, the link between employees’ CSR perception and OCB is well-documented in the prior literature (Ko et al., 2018; Oo et al., 2018). Further, in line with the work of Sen and Bhattacharya (2001) and Castro-González et al. (2019), the authors feel here that employees also evaluated their organization based upon its CSR engagement. When employees see their socially responsible organization shows an extra-commitment (voluntary) for the elevation of all stakeholders, they are self-motivated to support their organization. Thus, as an outcome of CSR, their advocacy behavior is formed.

Moreover, with regard to the theory of social identity, the advocacy behavior of employees is formed due to a social exchange mechanism with an organization as a social group. In this vein, CSR activities are attributed for a greater social benefit, thus employees may feel motivated to support their socially responsible organization. Buttressing this Rupp et al. (2013) acknowledged that CSR has every potential to meet the psychological needs of employees, driven by a social exchange mechanism. Thus a positive link between CSR and employee advocacy may be proposed:

*H1*: Theoretically, there may exist a positive association between CSR and employees’ advocacy behavior.

### Employee Engagement and CSR

Employee engagement has received significant attention in the prior literature to spur the extra-role performance of employees. For example, it was mentioned earlier in a plethora of studies that employee engagement is critical to foster the OCB of employees in an organization (Prabasari et al., 2018; Sugianingrat et al., 2019; Shams et al., 2020). At the same time, several other extra roles of employees including scouting behavior (Shore et al., 2006) and employee creativity (Mubarak and Noor, 2018). Given that an engaged employee is expected to show extra commitment to his organization, such employees willfully make extra efforts for the betterment of the organization. Moreover, engaged workers consider the organization not a place to provide them with paychecks and promotions, but they are emotionally associated with an organization (Saks, 2006). Considering the seminal importance of employee engagement, Kang and Sung (2017) showed that employee engagement can drive the positive communicating behavior, which is similar to advocacy behavior, of employees. More specifically, building on their work, recently, Lee (2021b) found a positive link between employee engagement and their advocacy behavior. Characterized by a deep level of enthusiasm and connectivity with the work, an engaged employee shows an extraordinary commitment to promoting his organization to the external community and acts as a defender (Men and Bowen, 2016). Stretching this, the work of Tsarenko et al. (2018) acknowledged engaged employees could show better advocacy behavior for their organizations. Therefore, it can be suggested that:

*H2*: Employees’ engagement with an organization can be positively linked with their advocacy behavior.

### CSR, Employee Engagement, and Advocacy Behavior

Considering the seminal importance of employees’ engagement for the success of an organization, it has been receiving considerable importance from contemporary scholars (Kaliannan and Adjovu, 2015). For example, Cesário and Chambel (2017) were convinced to realize the potential role of engaged employees for the success of an organization. At the same time, the studies have also reported that in a workplace with disengaged employees is hard to see any significant progress (Kim and Park, 2017; Kodden, 2020). Buttressing this, Chaudhary and Akhouri (2018a) posited that an engaged workforce shows an extra level of commitment to the success of an organization. Different factors drive employee engagement in a workplace. With this regard, the literature acknowledges CSR as a significant enabler to foster employee engagement (Gao et al., 2018). Specifically, it was reported in a study that CSR engagement of an organization was the third most preferred enabler to inculcate employees’ engagement (Perrin, 2007). The social exchange mechanism between employees and an organization due to CSR can significantly enhance their level of engagement (Gao et al., 2018; Nazir and Islam, 2020). The CSR engagement of a socially responsible organization helps employees to build a strong emotional bond on the part of employees. This strong emotional bond enhances their engagement with work (Mory et al., 2016). Responding to this, the study of Mirvis (2012) established a clear link between the CSR efforts of an organization and employees’ engagement. Moreover, referring to the theory of social identity, when employees feel trust and obligations with their ethical organization, such feelings spur their engagement. At the same time, the mediating role of employee engagement as an outcome of CSR is well recognized in the prior literature (Tian and Robertson, 2019; Raza et al., 2021; Wei et al., 2021). As engaged employees show better commitment to perform different extra roles in an organization, and CSR orientation of an organization has the potential to influence employees’ engagement, which can ultimately motivate employees to become advocates. Thus, the following hypotheses may be suggested.

*H3*: CSR commitment of an organization can positively induce employees’ engagement.

*H4*: Employees’ engagement mediates between CSR and employees’ advocacy behavior.

## Methodology

### Data Collection Process

The current work has selected the hotel sector of Pakistan. In this vein, it is to be noted that the hotel business in the country has a long history, as this sector has been operating in Pakistan for many decades. Currently, the hotel sector in the country represents a mixture of different national and international hotel chains. From the standpoint of the economy, the hotel sector has been contributing significantly to the gross domestic product (GDP) of Pakistan (more than 7% of total GDP), with almost a workforce of 4 million (Hadi, 2019). With the advancement in the country’s infrastructure and a special focus of the current government to promote tourism, the hotel sector in Pakistan has witnessed significant growth in recent years. It is also forecasted that the hotel business in Pakistan will likely receive an even better growth pace in the future.

The current study has focused on this sector for two reasons. First, as it was identified at the onset of this document that the hotel business is globally known for its out-sized turn-over, implying that the employees in this sector face a stressful situation (McNamara et al., 2011), which lowers their morale at work (Hotel Tech Report, 2020), thus it will be worthwhile to see whether CSR engagement of a hotel can raise the employees’ morale by enhancing their engagement. Second, with the rising competition in this sector, investigating employees’ advocacy behavior is also important because the information from a personal source is more trustworthy than the marketing-related communications provided by a hotel through different advertising media. Therefore, considering the importance of the above factors in this sector, the relevance of the current work with the hotel sector is not without logic.

Most of the large cities in Pakistan are famous for the hotel business. Currently, Avari, Marriot, Carlton, Regent, Pearl Continental, and Ramada Plaza international are some major international hotel chains operating in Pakistan. The authors targeted two large Pakistan cities, including Lahore and Islamabad, to collect the data for the current work. Given that both of these cities have a multi-million population and are famous for different tourist locations, almost all national and international hotel players operate in these cities. Prior to approaching a hotel with a request to participate in the current survey, different hotels were scrutinized by the authors to see if they were engaged in CSR activities or not. This scrutiny helped authors to identify a suitable list of hotels for the current survey. With this regard, it was realized that all large hotels were engaged in different CSR activities; however, only four hotels showed positive consent to facilitate the authors in the data collection activity.

The unit of analysis of the current survey were the individual employees serving in different hotels in Lahore and Islamabad. Specifically, employees from different departments and positions (managerial and non-managers) voluntarily participated in this survey. More specifically, given that Pakistan is a younger population with a mean age of 22.8 years, a representative sample between the ages of 18–40 and above was included in the survey. For more details, one can see Table 1.

**Table 1:** Demographic detail.

Demographic	Frequency	Percentage
**Gender**		
Male	247	67.67
Female	142	32.33
**Age**		
18–25	67	17.42
26–30	86	24.49
31–35	98	29.80
36–40	82	16.67
Above 40	56	11.62
**Experience**		
1–3	81	19.44
4–6	142	38.38
7–9	94	25.01
Above 10	72	17.17
**Category**		
Manager/supervisor	103	24.50
Non-manager	286	75.50

The data collection tool of the current survey was an adapted questionnaire which was finalized by including scales from different sources. The authors also requested the professionals from the field to assess the questionnaire before providing the questionnaire to the respondents. This expert opinion helped to verify the appropriateness of the questionnaires to serve the purpose of the current work (Gjersing et al., 2010; Fernández-Gómez et al., 2020). In general, the outlay of the questionnaire comprised two sections. The demographic information was requested in the first section, whereas, in the second section, the information related to the study’s constructs was obtained from the respondents. A total of 500 questionnaires (self-administered) were initially distributed among the employees of different hotels, who responded positively with a response rate of 78% (*n* = 389). Lastly, to maintain the ethical standards, the authors observed the ethical guidelines of the Helsinki Declaration.

### Measures

The constructs of the current work were operationalized by employing the scales from different sources. For example, the CSR scale was taken from the seminal work of Turker (2009). The original scale consisted of 17 items, however, the first 12 items were related to general CSR engagement and employee-related CSR activities of an organization. Generally, the literature suggests that employees’ behavior, especially their extra-role behavior is influenced by general CSR activities of an organization and employees’ related CSR policies. Under the domain of general CSR activities, the studies of Jahanshahi et al. (2021) and Ahmad et al. (2022) can be referred. These authors found that general CSR-related activities of an organization can boost the extra-role behavior of employees (advocacy is also an extra-role). Specifically, a recent research by Liu et al. (2022) indicates that employees’ CSR perceptions can drive their advocacy behavior. Similarly, under the domain of employees’ specific CSR the work of Hu et al. (2019) and Ahmad et al. (2021) can be cited. More specifically, the study of Lee (2021a) mentioned that internal CSR activities of an organization can urge employees to act as advocate for their organization. Thus the current study considered these 12 items to be included in the current survey to record the employees’ CSR perceptions. One sample item from general CSR engagement was “Our hotel participates to the activities which aim to protect and improve the quality of the natural environment,” whereas a sample item relevant to employees related CSR was “The management of our hotel primarily concerns with employees’ needs and wants.” The reliability value (*α*) of this scale was 0.948. In like vein, the construct of employees’ engagement—E.E was operationalized by employing the scale of Schaufeli et al. (2006). This is also a famous scale to record the employees’ perceptions of their work engagement. The scale contained nine items among which a sample item was, “I am proud of the work that I do.” The reliability value (*α*) of this scale was 0.931. Lastly, the construct of employees’ advocacy behavior—ADB was adapted from the work of Van Dyne et al. (1994). There were three items to capture the extent to which employees were willing to promote their hotel to the external community. One sample item from this scale was “I say positive things about my hotel to other people.” The reliability value (*α*) of this scale was 0.819. The responses were taken on a five-point Likert scale.

### Common Method Variance

The authors took different theoretical and empirical steps to address the potential issue of common method variance (CMV). Theoretically, the items of each construct were scattered on the questionnaire randomly. This step was helpful to mitigate any potential effort to build a sequence in answering the questions from a respondent. Additionally, the anonymity of each respondent was highly maintained as no such question was included, through which the identification of a respondent may be put at stake. Empirically, the authors carried out Harman’s single-factor test. To do this, SPSS software (version 23) was considered. In this vein, Principal Axis Factoring (PAF) was employed without using any rotation method. Further, the number of factors was set to “1.” Generally, the guideline to assess the result of single-factor lies in detecting a single factor that could explain 50% or more of the total variance. If such a factor exists, it implies that the data suffer from the issue of CMV. However, in the current case (Table 2), no such dominant single factor emerged, implying that the issue of CMV is not critical in the dataset of the current survey. At the same time, the authors also considered the technique of common latent factor (CLF) to cross verify the outcomes of Harman’s single factor. For this purpose, a measurement model was initially developed in AMOS software, which was then contrasted by introducing a CLF in the measurement model. The results again showed the CLF was not explaining any sheer amount of total variance.

**Table 2:** Results of single-factor analysis.

Factor	Initial Eigenvalues			Extraction sums of squared loadings		
Total	% of Variance	Cumulative %	Total	% of Variance	Cumulative %
1	10.595	44.145	44.145	10.173	42.387	42.387
2	1.890	7.875	52.020			
3	1.673	6.970	58.990			
4	1.384	5.767	64.757			
5	1.271	5.294	70.051			
6	1.185	4.937	74.988			
7	0.983	4.097	79.085			
8	0.774	3.224	82.309			
9	0.667	2.778	85.087			
10	0.585	2.439	87.526			
11	0.499	2.080	89.606			
12	0.427	1.778	91.384			
13	0.390	1.624	93.009			
14	0.298	1.242	94.250			
15	0.280	1.168	95.419			
16	0.237	0.987	96.406			
17	0.175	0.728	97.134			
18	0.160	0.667	97.801			
19	0.147	0.614	98.415			
20	0.105	0.437	98.852			
21	0.094	0.390	99.242			
22	0.086	0.358	99.600			
23	0.069	0.288	99.888			
24	0.027	0.112	100.000			

*Factoring method = Principal Axis Factoring*.

Moreover, the standardized regression weights of both measured models were also compared to detect any significant difference (a difference > 0.2). Such results have been reported in Table 3 for the readers. As it is evident from the result, the factor loadings of all the items did not change significantly in both cases (models with and without the CLF). All these results indicated that CMV if it existed in the current dataset, was not a critical issue.

**Table 3:** Common latent factor (CLF) results.

Item	Actual model	CLF model	Difference
CSR1←CSR	0.823	0.842	0.019
CSR2←CSR	0.817	0.829	0.012
CSR3←CSR	0.792	0.813	0.021
CSR4←CSR	0.733	0.762	0.029
CSR5←CSR	0.764	0.769	0.005
CSR6←CSR	0.729	0.741	0.012
ECP1←CSR	0.832	0.856	0.024
ECP2←CSR	0.811	0.822	0.011
ECP3←CSR	0.873	0.898	0.025
ECP4←CSR	0.914	0.916	0.002
ECP5←CSR	0.719	0.743	0.024
ECP6←CSR	0.728	0.751	0.023
E.E1←E.E	0.733	0.739	0.006
E.E2←E.E	0.749	0.758	0.009
E.E3←E.E	0.716	0.722	0.006
E.E4←E.E	0.893	0.898	0.005
E.E5←E.E	0.836	0.855	0.019
E.E6←E.E	0.712	0.741	0.029
E.E7←E.E	0.738	0.745	0.007
E.E8←E.E	0.846	0.862	0.016
E.E9←E.E	0.881	0.899	0.018
ADB1←ADB	0.868	0.872	0.004
ADB2←ADB	0.722	0.753	0.031
ADB3←ADB	0.844	0.856	0.012

## Results

### Construct Evaluation

To evaluate the constructs of the current survey (CSR, E.E, and ADB), different statistical tests were employed. For example, the factor loadings (standardized) of each construct were assessed, and it was found that no factor loading was less than 0.7, which shows each item’s factor loading (*λ*) was significant (Table 4). Moreover, the cases of cross-loadings were also non-evident in the dataset. Similarly, the convergent validity was also assessed for each construct. The authors calculated the average variance extracted (AVE) for all constructs separately in this vein. Usually, it is considered if the value of AVE for a construct is larger than 0.5, then it is assumed that the convergent validity is established (Fornell and Larcker, 1981). With this regard, all AVE values were found beyond 0.5 (CSR—0.635, E.E—0.628, and ADB—0.662). Therefore, it was assumed that all constructs qualified the condition of convergent validity. Lastly, the composite reliability (CR) was also calculated in each case, and it was revealed that the CR values for all constructs were significant (>0.7). For example, CR values for CSR, E.E, and ADB were 0.954, 0.938, and 0.854, respectively.

**Table 4:** Outputs of construct evaluation.

Construct	Λ	*λ* ^2^	E-variance	∑*λ*^2^	Items	AVE	CR
CSR	0.823	0.677	0.323				
	0.817	0.667	0.333				
	0.792	0.627	0.373				
	0.733	0.537	0.463				
	0.764	0.584	0.416				
	0.729	0.531	0.469				
	0.832	0.692	0.308				
	0.811	0.658	0.342				
	0.873	0.762	0.238				
	0.914	0.835	0.165				
	0.719	0.517	0.483				
	0.728	0.530	0.470	7.619	12	0.635	0.954
Engagement	0.733	0.537	0.463				
	0.749	0.561	0.439				
	0.716	0.513	0.487				
	0.893	0.797	0.203				
	0.836	0.699	0.301				
	0.712	0.507	0.493				
	0.738	0.545	0.455				
	0.846	0.716	0.284				
	0.881	0.776	0.224	5.651	9	0.628	0.938
Advocacy behavior	0.868	0.753	0.247				
	0.722	0.521	0.479				
	0.844	0.712	0.288	1.987	3	0.662	0.854

**λ*, item loadings, CR, composite reliability, ∑*λ*^2^, sum of square of item loadings, and E-variance, error variance*.

### Correlations

The results of correlation analysis have been reported in Table 5. According to these results, the correlation values (*r*) were all positive in each case. For instance, the values of r for CSR <=> E.E, and CSR <=> ADB were 0.339, and 0.523, respectively. These cases showed that the constructs were positively correlated with one and others. Moreover, r values in each case were modest (not beyond 0.7), implying that there was no issue of multi-collinearity. Additionally, the authors also developed different measurement models (hypothesized vs. alternate). These models were then assessed for their superiority based on different model fit values, including normed fit index (NFI), comparative fit index (CFI), root mean square error of approximation RMSEA, and chi-square values (*χ*^2^). Table 6 includes the results of these alternate and hypothesized models. In this regard, it was found that the hypothesized three-factor-mediated model (model-1) produced superior values in every case, implying that there was a good fit between theory and the data compared to the alternate models.

**Table 5:** Correlations and discriminant validity.

Construct	CSR	E.E	ADB	Mean	SD
CSR	**0.797**	0.339^**^	0.523^**^	3.06	0.66
E.E		**0.792**	0.413^**^	2.89	0.74
ADB			**0.814**	2.96	0.69

*SD, standard deviation*.

** *= significant values of correlation, bold diagonal = discriminant validity values*.

**Table 6:** Model fit comparison hypothesized vs. alternate models.

	Model-1 (Hypothesized)	Model-2 Two-factor	Model-3 Three factor
*χ*^2^ (*df*)	1142.063 (847)	1723.866 (562)	1488.729 (719)
*χ*^2^/*df*	1.348	3.525	2.070
NFI	0.961	0.838	0.892
CFI	0.969	0.874	0.919
RMSEA	0.0342	0.063	0.055

### Hypotheses Evaluation

In the last place of the data analysis phase, the authors validated the hypotheses of the current study. In doing so, the structural model was developed twice. Firstly, the structural model was developed to see the direct effects on ADB without considering the mediating role of E.E. This model was developed to validate the first three hypotheses of the current work (H1, H2, and H3). The outputs of the direct effect structural model have been presented in Table 7. As per the results, it can be seen that the first three hypotheses were significant, and hence these were accepted. To explain further, the beta values (*β*), CI, and *p* values were assessed. It was observed that all *p* values were significant, and CI did not include a zero-value in any case. Moreover, *β-*values were all positive in all three cases (CSR→ADB = 0.542; E.E→ADB = 0.428; and CSR→E.E = 0.367). To conclude, H1, H2, and H3 were accepted.

**Table 7:** Outputs of direct effect model.

Path	Relation	Estimates	SE	CR	*p*-value	CI-range	Decision
CSR→ADB (H1)	+	(β1) 0.542^**^	0.039	13.897	***	0.261 – 0.249	Accepted
E.E→ADB (H2)	+	(β2) 0.428^**^	0.052	8.231	***	0.239 – 0.218	Accepted
CSR→E.E (H3)	+	(β3) 0.367^**^	0.058	6.327	***	0.176 – 0.163	Accepted

*CI, confidence interval*.

** *= significant values, SE = standard error, and + = positive relationship;*

*** = significant values, SE = standard error, and + = positive relationship.

Secondly, the structural model was developed to record the mediating effect of E.E (H4). To do this, the bootstrapping method was considered by the authors by using a larger bootstrapping sample of 2,000 to validate the mediating effect of E.E. The results of this mediated structural model have been presented in Table 8 which shows that E.E partially mediates between CSR and ADB (CSR→E.E→ADB = 0.157). The same criterion (stated above) was employed to reach such results, and it was found that all values were significant. Therefore, the mediating role of E.E was confirmed, and thus H4 of the current study was accepted.

**Table 8:** Mediation analysis.

Path	Relation	Estimates	SE	Z-score	*p*-value	CI-range	Decision
CSR→E.E→ADB (H4)	+	(β4) 0.157^**^	0.028	5.607	***	0.093 – 0.087	Accepted

*CI, confidence interval*.

** *= significant values, SE = standard error, and + = positive relationship;*

*** = significant values, SE = standard error, and + = positive relationship.

## Discussion

There were some specific objectives to carry out the current work, which can now be discussed in detail, followed by the statistical results. Firstly, it was realized that the CSR engagement of a hotel could positively induce the employees’ psychology by converting them into advocates. At one end, employees positively evaluate their socially responsible hotel’s CSR activities. At the other end, they are self-convinced to respond positively by supporting their hotel through their extra-role engagement. One such extra-role includes employees’ advocacy behavior. Given that there has been mounting importance among contemporary scholars regarding CSR perceptions of employees. Moreover, the recent shift in the field of CSR from a meso level to a micro-level (at an individual level) also indicates the importance of CSR from the perspective of employees’ perceptions. Earlier research also showed that employees’ CSR perception could influence employees’ behavior through the sense-making of their organization’s CSR commitment (Glavas, 2016; Vlachos et al., 2017; Hur et al., 2021). Specifically, the current work’s findings enrich the readers’ understanding of how CSR works rather than focusing on whether it works or not (Barnett and Salomon, 2012). Importantly, the current research tries to explain the underlying mechanism of how employees’ advocacy behavior can be spurred as an outcome of CSR.

Secondly, the current analysis results also showed that employees’ engagement could mediate CSR and employees’ advocacy behavior. Although the mediating potential of employees’ engagement as an antecedent of CSR was already established in the prior literature (Chaudhary and Akhouri, 2018b; Ali et al., 2020), its potential role to induce employees’ advocacy behavior was neglected. With this regard, the current study’s results showed that employees’ CSR perceptions about a socially responsible hotel help them induce their level of engagement, which then induces their advocacy behavior. Prior research has also acknowledged that engaged employees are more committed to supporting their organization by performing different voluntary tasks (Song et al., 2012; Demerouti et al., 2015). Moreover, the theory of social identity also provides the logic of the above outcomes. As the employees strongly identify themselves with an organization due to its social engagement, this strong identification motivates every employee to put forth every effort which can benefit their social group’s performance. In the current context, CSR perceptions of employees can lead the employees toward a higher level of engagement, and engaged workers are better suited to be converted as advocates.

### Implications for Theory

The current study enriches the literature in three ways. In the first place, considering the mounting importance of CSR at the micro-level, the current work offers a unique direction by proposing employees’ CSR perceptions as a motivator to enhance their advocacy. Though the domain of micro-CSR is receiving considerable academic attention, previously, the prime focus of such research studies was the pro-environmental behavior of employees (Ahmad et al., 2021; Yu et al., 2021) or their citizenship behavior (Ong et al., 2018). In this regard, the current study offers a different CSR perspective, which was not well-explored previously.

In the second place, the current study is one of the sparse studies that note the mediating potential of employees’ engagement between the relationship of CSR and employees’ advocacy behavior in a unified model. Given that organizational and personal factors influence the employees’ behavior, the current work attempts to consider both of these factors to shape employees’ advocacy behavior. For instance, at an organizational level, CSR perceptions of employees were considered, and at a personal level, their engagement was taken into account. The authors feel that considering both factors can well explain the underlying mechanism due to which employees become advocates for their socially responsible hotel. In the last place, the current work advances the literature of the hospitality sector from the perspective of CSR and advocacy behavior. Given that this sector has been largely reported for its high employee turnover (Glenn, 2016; Erica, 2019; Amanda, 2020), and stiff rivalry, the current work attempts to help this sector by proposing CSR for a win-win strategy by fostering employees’ engagement and advocacy behavior.

### Implications for Practice

When looked at from the lens of practical implications, the current work is equally important as it offers different practical implications to the hotel sector of Pakistan. First of all, the current work offers a different insight into hotel enterprises’ management to foster employees’ engagement to improve their advocacy behavior through CSR. As mentioned earlier, the hotel sector is badly reputed globally for a higher turnover and disengaged workers, the above finding has a special significance to this sector. In this vein, the current study offers this sector an effective tool in the form of CSR to keep the employees well-engaged and motivated to perform different voluntary tasks, including their advocacy role.

Likewise, from the standpoint of rivalry in this sector, the insights of the current study are of much importance. Considering the importance of personal sources of information, compared to the commercial sources launched by a hotel, the advocacy behavior of employees, mainly driven by the CSR perceptions of employees, can lead a hotel to outperform its rivals. Additionally, with regard to service-dominant logic, the role of employees for services is critical compared to the manufacturing sector. Therefore, the advocacy behavior of employees not only helps a hotel improve its reputation but also motivates the employees to deliver superior services for their socially responsible hotel. Lastly, employees being the stakeholders perceive their organization as “one of us,” thus they can serve as credible organizational spokespersons who could promote an organization, externally.

### Limitations and Future Research Directions

Like in all cases, the current work is not without limitations, however, the authors feel such limitations can lead future researchers toward new arenas for CSR-advocacy relationship. In this vein, the data were collected from a single source, implying that elimination of CMV may be difficult. This limitation may be addressed in future studies by employing an experimental research design and by collecting data from multiple sources. Similarly, another limitation of the current work is explaining employee behavior through CSR and employees’ engagement. Although the proposed relations were significant, considering the complex nature of human behavior, more constructs may be included in the current framework. For example, employees’ desire for volunteerism may also be considered as an important moderator. Similarly, given that the data of the current work was cross-sectional, it undermines the causal relations among the constructs. Therefore, it is desirable to employ a longitudinal data collection technique in future researches. Lastly, it would be interesting for the future researchers to investigate if a rival organization has a better CSR strategies, will it create poaching or attrition effect on employees.

## Conclusion

In conclusion, the current work helps the hotel sector of Pakistan by promoting employees’ advocacy behavior which is undoubtedly is of paramount importance for any hotel. In this vein, the management of the hotel is suggested to develop CSR strategies aligned with the mission and vision of a hotel. At the same time, the management should emphasize on employees to realize the CSR activities of a socially responsible hotel as value-driven. For the hotel sector, to have a sustainable management philosophy, it is important to take the employees on board by communicating effectively about the concern of a hotel for social benefits. On a further note, the management should realize that employees evaluate CSR engagement of a hotel as a benefit for all stakeholders, and being an important stakeholder, they are urged to respond to their socially responsible hotel positively by acting as advocates.

## Data Availability Statement

The raw data supporting the conclusions of this article will be made available by the authors, without undue reservation.

## Author Contributions

NA, ZU, EA, HH, AA-M, and AV-M contributed to conceptualization, formal analysis, investigation, methodology, and writing and editing of the original draft. All authors contributed to the article and approved the submitted version.

## Conflict of Interest

The authors declare that the research was conducted in the absence of any commercial or financial relationships that could be construed as a potential conflict of interest.

## Publisher’s Note

All claims expressed in this article are solely those of the authors and do not necessarily represent those of their affiliated organizations, or those of the publisher, the editors and the reviewers. Any product that may be evaluated in this article, or claim that may be made by its manufacturer, is not guaranteed or endorsed by the publisher.
